This article has been retracted.

# miR-152-3p Affects the Progression of Colon Cancer via the KLF4/IFITM3 Axis

**DOI:** 10.1155/2020/8209504

**Published:** 2020-09-01

**Authors:** Xiaoyi Zhu, Zhan Shen, Da Man, Hang Ruan, Sha Huang

**Affiliations:** ^1^Department of Colorectal Surgery, Shulan (Hangzhou) Hospital, Hangzhou 310000, China; ^2^Department of Plastic Surgery, Shulan (Hangzhou) Hospital, Hangzhou 310000, China

## Abstract

**Objective:**

The purpose of this study was to investigate the relationship between miR-152-3p and the KLF4/IFITM3 axis, thereby revealing the mechanism underlying colon cancer occurrence and development, consequently providing a promising target for colon cancer treatment.

**Methods:**

Bioinformatics methods were implemented to analyze the differential expression of miRNAs and mRNAs in colon cancer, confirm the target miRNA, and predict the downstream targeted mRNAs. qRT-PCR and Western blot were performed to detect the expression of miR-152-3p, KLF4, and IFITM3. CCK-8 and colony formation assays were conducted for the assessment of cell proliferation, and flow cytometry was carried out for the detection of cell apoptosis. Finally, dual-luciferase reporter gene assay was employed to verify the targeting relationship between miR-152-3p and KLF4.

**Results:**

miR-152-3p was highly expressed in colon cancer cells, whereas KLF4 was poorly expressed. Dual-luciferase assay verified that miR-152-3p targeted to bind to KLF4 and suppressed its expression. Moreover, silencing miR-152-3p or overexpressing KLF4 was found to downregulate IFITM3, thereby inhibiting cell proliferation and potentiating cell apoptosis. In rescue experiments, we found that miR-152-3p deficiency decreased the expression of IFITM3 and weakened cancer cell proliferation, and such effects were restored when miR-152-3p and KLF4 were silenced simultaneously.

**Conclusion:**

In sum, we discovered that miR-152-3p can affect the pathogenesis of colon cancer via the KLF4/IFITM3 axis.

## 1. Introduction

Colon cancer is the fourth common malignant tumor worldwide and the fifth cause of cancer-related deaths, with confirmed cases around 1,096,601 in 2018 and deaths up to 551,269 1. Due to the change in people's lifestyle and diet, the morbidity of colon cancer annually increases, and the age of people suffering from this cancer tends to be lower, leading to a high rank (3^th^) among gastrointestinal malignancies in China 2. Therapies currently for colon cancer mainly include surgical resection, chemotherapy, radiotherapy, and targeted therapy-based comprehensive treatment 3, but the efficacy in advanced patients remains poor with clinical symptoms partially relieved 4. Statistically, for the patients with no metastasis, with local metastasis, and with distant metastasis, their 5-year survival rate was 90%, 70%, and 10%, respectively 5. Thus, exploring biomarkers for early diagnosis of colon cancer and therapeutic targets is beneficial for better treatment and prognosis.

KLF4 (Kruppel-like factor 4), a zinc finger transcription factor, is involved in the regulation of thymocyte as well as the colonic goblet cell proliferation, differentiation, apoptosis, and metabolism 6, 7. Studies have proved that KLF4 is differentially expressed in various human cancers, such as prostate cancer 8, liver cancer 9, and breast cancer 10. In addition, KLF4 has been considered as a molecular target that can be used in cancer treatment. For example, FBXO32 can promote the degradation of the KLF4 proteasome to suppress the occurrence of breast cancer 11. In hepatocellular carcinoma, KLF4 can function on cell growth and migration via the CDH3/GSK-3*β* axis 12, while in colon cancer KLF4 is always reported acting as an oncogene. Decreased KLF4 was observed to inhibit NDRG2 signal-dependent cell proliferation in colorectal cancer, which provides a theoretical basis for early diagnosis and treatment 13. Moreover, KLF4 can enhance the sensitivity of colon cancer cells to cisplatin through altering the expression of HMGB1 (high-mobility group box 1) and hTERT (human telomerase reverse transcriptase) 14. Another study also found that IFITM3 is a direct transcription target of KLF4 in colon cancer, and decreased KLF4 leads to the upregulation of IFITM3, thereby promoting progression and metastasis 15.

In the present study, we predicted that there were targeted binding sites of miR-152-3p on KLF4 3′UTR and found that miR-152-3p was highly expressed in colon cancer, which has never been reported. In view of this, we made further efforts and confirmed that miR-152-3p targeted KLF4 to mediate the expression of IFITM3 and affect the development of colon cancer.

## 2. Materials and Methods

### 2.1. Bioinformatics Analysis

Expression profiles of mRNAs and miRNAs associated with colon cancer were obtained from TCGA database (https://portal.gdc.cancer.gov/). “edgeR” package was employed to perform differential analysis (∣log FC | >2, *p*adj < 0.05) to find the differentially expressed miRNAs (DEmiRNAs), which were subjected to survival analysis combined with the matched clinical information. Three databases miRDB (http://mirdb.org/), miRTarBase (http://mirtarbase.mbc.nctu.edu.tw/php/index.php), and TargetScan (http://www.targetscan.org/vert_71/) were applied to predict the targets of the target miRNA. Venn diagram was plotted to find the candidate targeted mRNAs.

### 2.2. Cell Culture

Human normal colon cell line CCD-18Co (BNCC337724), human embryonic kidney cell line HEK-293T (BNCC338274), and colon cancer cell lines HT29 (ATCC HTB-38), HCT116 (BNCC337692), and SW480 (BNCC100604) were all purchased from the American Type Culture Collection. All cells were grown in Dulbecco's Modified Eagle's Medium (DMEM; Gibco, Thermo Fisher Scientific, Inc., Waltham, MA, USA) containing 10% fetal bovine serum (FBS; HyClone; GE Healthcare Life Sciences, Logan, UT, USA) and 100 U/mL streptomycin/penicillin (Gibco; Thermo Fisher Scientific, Inc.) and maintained in 5% CO_2_ at 37°C. Mediums were replaced every 2 or 3 days.

### 2.3. Cell Transfection

miR-152-3p mimic, miR-152-3p inhibitor, si-KLF4, and their negative controls (mimic NC, inhibitor NC, and si-NC) were purchased from GenePharma (Shanghai, China). Overexpression plasmids targeting KLF4 and IFITM3 (oe-KLF4 and pre-IFITM3) and their negative controls (oe-NC and pre-NC) were ordered from Miaoling Biotechnology (Wuhan, China). For transfection, Lipofectamine 2000 (Thermo Fisher Scientific, Inc.) was used following the manufacturer's instructions. Transfected cells were maintained in DMEM containing 5% CO_2_ at 37°C for subsequent experiments. All cells grew in complete mediums for at least 24 h and were washed in PBS (pH 7.4) before transfection.

### 2.4. qRT-PCR

Total RNA was extracted using TRizol (Invitrogen), treated by DNase I (TaKaRa) for the removal of the genomic DNA, and then reversely transcribed into cDNA by reverse transcriptase M-MLV (TaKaRa). Applied Biosystems 7300 Real-Time PCR System (Applied Biosystems, USA) was employed to test the KLF4 mRNA expression, and the result was expressed in 2^-*ΔΔ*Ct^. Primer sequences were as follows: KLF4-F: 5′-ATGGCTGTCAGCGACGCGCTGC-3′, KLF4-R: 5′-TTAAAAATGCCTCTTCATGTGTAAGGCG-3′; GAPDH-F: 5′-GCACCGTCAAGCTGAGAAC-3′, GAPDH-R: 5′-TGGTGAAGACGCCAGTGGA-3′.

RNAiso technology (TaKaRa, Dalian, China) was applied to isolate the total RNA from cancer cells and solid tumors. The expression of miR-152-3p was analyzed by a TaqMan RT kit (Applied Biosystems) and TaqMan MicroRNA kit (Applied Biosystems) under the Applied Biosystems 7300 Real-Time PCR System (Applied Biosystems, USA), and 2^-*ΔΔ*Ct^ was performed to normalize the miR-152-3p expression. The primers were designed as follows: miR-152-3p-F: 5′-ACACTCCAGCTGGGTCAGTGCATGACAG-3′, miR-152-3p-R: 5′-CTCAACTGGTGTCGTGGAGTCGGCAATTCAGTTGAGCCAAGTT-3′; U6-F: 5′-GCTTCGGCAGCACATATACTAAAAT-3′, U6-R: 5′-CGCTTCAGAATTTGCGTGTCAT-3′.

### 2.5. Western Blot

After 48 h of transfection, cells were washed in cold PBS for three times and then lysed on ice with whole cell lysate for 10 min, with the concentration of the product sequentially determined using the BCA protein assay kit (Thermo Fisher Scientific, Waltham, MA, USA). Subsequently, 30 *μ*g of the total proteins was separated by polyacrylamide gel electrophoresis (PAGE) and then transferred onto polyvinylidene fluoride (PVDF) membranes (Amersham, USA). After being blocked in 5% skim milk at room temperature for 1 h, the membranes were incubated overnight at 4°C with primary antibodies, followed by horseradish peroxidase- (HRP-) labeled secondary antibody goat anti-rabbit IgG H&L (ab6721, 1 : 2000, Abcam, Cambridge, UK) at room temperature for 1 h. Primary antibodies included KLF4 rabbit polyclonal antibody (ab215036, 1 : 1000, Abcam, Cambridge, UK), IFITM3 rabbit polyclonal antibody (ab109429, 1 : 1000, Abcam, Cambridge, UK), and GAPDH rabbit polyclonal antibody (ab9485, 1 : 2500, Abcam, Cambridge, UK). PBST (PBS buffer containing 0.1% Tween-20) was used to wash the membranes after each reaction. An optical luminometer (GE, USA) was employed to visualize the protein bands.

### 2.6. Dual-Luciferase Reporter Gene Assay

Amplified wild-type (WT) and mutant (MUT) KLF4 3′UTR were inserted into the pMIR reporter vectors (Ambion; Thermo Fisher Scientific, Inc.). Constructs WT-KLF4 and MUT-KLF4 were cotransfected with the miR-152-3p mimic/miR-152-3p inhibitor or their negative controls into HEK-293T cells (BNCC338274), respectively. The Renilla luciferase vector pRL-TK (TaKaRa, Dalian, China) was taken as the internal reference. The luciferase activity was assayed by a luciferase reporter kit (Promega, Madison, WI).

### 2.7. CCK-8

96-well plates were used for cell culture at a density of 1 × 10^4^ cells/well. The specific procedures proceeded as previously described 16. According to the protocols of the CCK-8 kit (Dojindo, Japan), cell viability was examined at 0, 24, 48, and 72 h, respectively. The absorbance at 450 nm in wavelength of each well was read.

### 2.8. Colony Formation Assay

Transfected cells were seeded into 6-well plates (1 × 10^3^ cells/well) and cultured in DMEM supplemented with 10% FBS at 37°C. After two weeks, the cells were washed in PBS, fixed with 10% formalin, and stained by 0.1% crystal violet (Sigma, USA). Cell colonies that were visible to the naked eyes were counted at the end.

### 2.9. Flow Cytometry

Annexin V and Propidium Iodide (PI) fluorescein staining kits (Bender MedSystems, Austria) were applied in this experiment. 5 × 10^5^ cells were suspended in 500 *μ*L (1x) binding buffer (10 mM HEPES pH 7.4, 140 mM NaCl, and 2.5 mM CaCl_2_) for preparation. Then, the cell suspension was incubated with Annexin V (1 : 20) for 5 min, followed by PI for another 15 min. Cell apoptosis was analyzed by flow cytometry, and cell apoptotic rate was calculated.

### 2.10. Statistical Analysis

All data were processed by the SPSS 22.0 software (SPSS Inc., Chicago, IL, USA) and GraphPad Prism 6.0 software (GraphPad Prism 6.0; San Diego, CA, USA). Mean ± standard deviation (SD) was used to express the measurement data, while *t* test and one-way ANOVA were performed to analyze the differences between two groups and among multiple groups. All results were representative of at least three independent experiments. *p* < 0.05 was considered statistically significant.

## 3. Results

### 3.1. Bioinformatics Analysis

In all, 239 DEmiRNAs (Figure 1(a)) and 2065 DEmRNAs (Figure 1(b)) were obtained by differential analysis. Among the DEmiRNAs, 4 miRNAs (miR-145, miR-152, miR-193b, and miR-216a) with survival significance were screened, of which miR-152 exhibited a significant correlation with the survival of colon cancer (Figure 1(c)) and was remarkably elevated in the colon cancer tissue (Figure 1(e)). Relevant literature reported that miR-152 is involved in the ceRNA network 17. Thus, miRDB, miRTarBase, and TargetScan databases were used to predict the targets for miR-152, and eventually, 68 targeted mRNAs were obtained. Thereafter, 4 candidate mRNAs, including KLF4, BMP3, NPTX1, and ARID3A (Figure 1(d)), were identified from the intersection of these predicted mRNAs and downregulated DEmRNAs in TCGA. KLF4, which was observed to be significantly decreased in the cancer tissue in TCGA-COAD dataset, was selected for follow-up analysis (Figure 1(f)).

### 3.2. miR-152-3p Is Highly Expressed in Colon Cancer Cells and Affects the Proliferation and Apoptosis of Cancer Cells *In Vitro*

In order to further investigate the role of miR-152-3p in colon cancer, qRT-PCR was primarily conducted to examine the expression of miR-152-3p in tumor cells (Figure 2(a)). It turned out that the miR-152-3p expression was significantly elevated in the cancer cell lines HT29, HCT116, and SW480 relative to that in the normal cell line CCD-18Co. Hence, the HT29 cell line where miR-152-3p was most highly expressed was selected for follow-up analysis.

miR-152-3p mimic, miR-152-3p inhibitor, and their negative controls were transfected into HT29 cells, respectively. Transfection efficiency was detected by qRT-PCR, and it was found that miR-152-3p was remarkably overexpressed or silenced in cells transfected with miR-152-3p mimic or inhibitor (Figure 2(b)). Thereafter, CCK-8 and colony formation assays were performed for the examination of cell proliferation. As shown in Figures 2(c) and 2(d), cells transfected with miR-152-3p mimic had an increased cell viability and stronger colony-forming ability, whereas cells with low miR-152-3p expression were accompanied with a reduced cell proliferation. Moreover, as revealed by flow cytometry, miR-152-3p silencing greatly increased cell apoptosis (Figure 2(e)).

### 3.3. Overexpression of KLF4 Mediates IFITM3 to Suppress the Proliferation of Colon Cancer Cells

KLF4 as a potential target of miR-152-3p is worthy of further exploration. Published literature reported that KLF4 can negatively mediate IFITM3 and plays a crucial role in the pathogenesis of colon cancer 15. Therefore, we firstly carried out qRT-PCR to detect the expression of these two genes in colon cancer cell lines. Compared with normal cells, KLF4 was significantly downregulated in colon cancer cells, while IFITM3 was upregulated (Figure 3(a)). Subsequently, Western blot was used to assess the protein levels of KLF4 and IFITM3 in cells transfected with oe-NC+pre-NC, oe-KLF4+pre-NC, and oe-KLF4+pre-IFITM3, finding that IFITM3 was greatly decreased in the oe-KLF4+pre-NC group by comparison with the oe-NC+pre-NC group (Figure 3(b)).

Moreover, the KLF4 overexpression was found to reduce cell viability and colony-forming ability as well as promote cell apoptosis, yet such effects were reversed upon the cooverexpression of KLF4 and IFITM3 (Figures 3(c)–3(e)). Collectively, it elucidated that KLF4 could function on the progression of colon cancer by regulating the expression of IFITM3, and its inhibitory effect on cancer cells could be suppressed with the upregulation of IFITM3.

### 3.4. KLF4 Is a Direct Target of miR-152-3p

As mentioned above, we predicted that miR-152-3p might target to regulate KLF4 (Figure 4(a)). To deeply explore the relationship between miR-152-3p and KLF4, dual-luciferase reporter gene assay was conducted, demonstrating that the markedly decreased luciferase activity happened in cells transfected with miR-152-3p mimic and WT-KLF4, while the highest activity occurred in cells with the miR-152-3p inhibitor and WT-KLF4 (Figure 4(b)). Western blot showed that the miR-152-3p overexpression reduced the KLF4 protein level but elevated the IFITM3 protein expression (Figure 4(c)).

### 3.5. miR-152-3p Affects Colon Cancer Cell Growth via Regulating the KLF4/IFITM3 Axis

To validate the regulation of miR-152-3p on KLF4/IFITM3 and clarify the role of such regulation in colon cancer, rescue experiment was carried out. Inhibitor NC+si-NC, miR-152-3p inhibitor+si-NC, and miR-152-3p inhibitor+si-KLF4 were used to transfect cells. As plotted in Figure 5(a), KLF4 was greatly upregulated when miR-152-3p was inhibited, whereas IFITM3 was significantly downregulated. Notably, the IFITM3 protein level was recovered near to the level in the inhibitor NC+si-NC group when miR-152-3p and KLF4 were silenced concurrently. In addition, CCK-8 and colony formation assays revealed that the low miR-152-3p expression repressed cell viability and colony-forming ability, but such inhibitory effect was reversed after KLF4 was silenced (Figures 5(b) and 5(c)). Moreover, in agreement with the results concluded above, increased KLF4 indicated a high apoptosis rate, as shown in Figure 5(d).

## 4. Discussion

In our study, we first confirmed that miR-152-3p was highly expressed in colon cancer cells, and silencing miR-152-3p could inhibit cell proliferation and growth. Also, we found that KLF4 was a direct target of miR-152-3p by conducting bioinformatics methods and dual-luciferase reporter gene assay. Finally, we used various experiments and elucidated a miR-152-3p-dependent mechanism by which miR-152-3p affected colon cancer cell proliferation and growth via the KLF4/IFITM3 axis.

MicroRNAs (miRNAs) can promote the degradation and inhibit the translation of mRNAs by interacting with 3′UTR of the target genes in eukaryotic cells, thereby participating in gene regulation in the posttranscriptional level 18. Being able to be expressed in various malignancies 19, miRNAs can not only serve as protooncogenes 20, 21 but also act as tumor suppressor genes affecting tumorigenesis and cancer cell differentiation 22. In diverse cancer tissues and cells, miR-152-3p exhibits significantly different expression levels. For instance, in breast cancer, the upregulation of miR-152-3p exerts its antitumor role by negatively regulating PIK3CA to suppress the activation of AKT and RPS6, thus inhibiting the HCC1806 cell proliferation 23. However, in glioma 24 and leukemia 25, the expression of miR-152-3p was reported to be elevated in cancer tissue and cells, which is significantly higher than that in normal tissue and cells. Interestingly, there is a study revealing that miR-152-3p is differentially expressed in different T_stages (T1-T4) of colon cancer, with increased expression in T2-T4 and relatively higher expression in T2 and T4 26. In this study, bioinformatics analysis and qRT-PCR revealed that miR-152-3p was markedly elevated in colon cancer tissue and cells, and silencing miR-152-3p led to decreased cell proliferation but increased cell apoptosis.

KLF4 is a transcription factor belonging to the Kruppel-like family and mediates some basic biological progresses, such as cell proliferation, differentiation, and migration 27. KLF4 is highly expressed in colon cells, especially in well-differentiated cells 28. In our research, KLF4 was verified to be significantly downregulated in colon cancer cells. Additionally, when KLF4 was overexpressed, cancer cell proliferation was greatly repressed, indicating the antitumor role of KLF4 overexpression in colon cancer. Some literatures have reported underlying mechanisms of KLF4 in cancers. For example, miR-10b mediates colorectal cancer cell metastasis and proliferation via targeting KLF4 29, which is consistent with our study. Furthermore, high KLF4 expression plays an inhibitory role in colon cancer development through suppressing IFITM3, which is an interferon-inducible gene overexpressed in colorectal cancer 15. In the present study, we conducted Western blot to assay the protein expression of IFITM3 and also found that IFITM3 was significantly downregulated with the presence of KLF4 overexpression.

Furthermore, targeted binding sites of miR-152-3p on KLF4 were predicted through bioinformatics methods, and miR-152-3p was verified to suppress KLF4 via qRT-PCR and Western blot. Dual-luciferase reporter gene assay indicated that KLF4 was a direct target of miR-152-3p, and that was in agreement with the report on glioma 24. In the cell level, we found that silencing miR-152-3p was observed to potentiate the synthesis of the KLF4 protein, resulting in the inhibition of cell proliferation and the promotion of apoptosis. Moreover, the trend of the expression of miR-152-3p and IFITM3 was demonstrated to be consistent. Rescue experiments elucidated that the expression of IFITM3 was remarkably restored when miR-152-3p and KLF4 were simultaneously silenced, indicating that miR-152-3p might affect the IFITM3 expression by targeting KLF4, thus regulating colon cancer cell proliferation and growth.

In conclusion, our study explored a miR-152-3p-dependent mechanism by which miR-152-3p affects colon cancer progression via the KLF4/IFITM3 axis, which was never studied before. Our findings provide potent reference for the molecular targeted therapy towards colon cancer.

## Figures and Tables

**Figure 1:** Bioinformatics analysis. Volcano plots were made to find the (a) DEmiRNAs and (b) DEmRNAs in TCGA-COAD dataset. (c) Survival analysis was performed, and it was found that miR-152-3p was of remarkable survival significance. (d) Venn diagram was plotted to find the candidate target genes from the predicted mRNAs of miR-152-3p and the DEmRNAs in TCGA-COAD dataset. (e) miR-152-3p was shown to be significantly upregulated in the colon cancer tissue in TCGA-COAD dataset. (f) KLF4 was verified to be noticeably lowly expressed in cancer tissue in TCGA-COAD dataset.

**Figure 2:** miR-152-3p is upregulated in colon cancer cells and affects cancer cell proliferation and apoptosis. miR-152-3p was significantly increased in (a) colon cancer cell lines HT29, HCT116, and SW480 relative to the normal cell line CCD-18Co. (b) qRT-PCR, (c) CCK-8, (d) colony formation assay, and (e) flow cytometry were conducted to assess the expression of miR-152-3p, cell viability, colony-forming ability, and apoptosis in each treatment group (∗ means *p* < 0.05).

**Figure 3:** The overexpression of KLF4 mediates the IFITM3 expression to regulate colon cancer cell proliferation and apoptosis. (a) The expression of KLF4 and IFITM3 in the normal cell line CCD-18Co and colon cell lines HT29, HCT116, and SW480 was detected by qRT-PCR. (b) Western blot was carried out for the protein examination of KLF4 and IFITM3 in cells transfected with oe-NC+pre-NC, oe-KLF4+pre-NC, and oe-KLF4+pre-IFITM3. (c) CCK-8, (d) colony formation assay, and (e) flow cytometry were performed to determine cell viability, colony-forming ability, and cell apoptosis (∗ means *p* < 0.05).

**Figure 4:** miR-152-3p targets KLF4 and decreases its expression. (a) Binding sites of miR-152-3p on KLF4 3′UTR were predicted by the bioinformatics method. (b) Dual-luciferase assay was done for the validation of the targeting relationship between miR-152-3p and KLF4. (c) Western blot was conducted to test the protein expression of KLF4 and IFITM3 in each treatment group (∗ means *p* < 0.05).

**Figure 5:** miR-152-3p affects colon cancer cell proliferation and apoptosis via the KLF4/IFITM3 axis. (a) Western blot was carried out to determine the protein expression of KLF4 and IFITM3 in cells transfected with inhibitor NC+si-NC, miR-152-3p inhibitor+si-NC, and miR-152-3p inhibitor+si-KLF4. (b) CCK-8, (c) colony formation assay, and (d) flow cytometry were conducted to assay cell viability, colony-forming ability, and apoptosis in each treatment group (∗ means *p* < 0.05).

## Data Availability

The data used to support the findings of this study are included within the article. The data and materials in the current study are available from the corresponding author on reasonable request.
